The article "Network Pharmacology and Bioinformatics Methods Reveal the Mechanism of Berberine in the Treatment of Ischaemic Stroke" was published in 2022. Journal: Evid Based Complement Alternat Med.

# Network Pharmacology and Bioinformatics Methods Reveal the Mechanism of Berberine in the Treatment of Ischaemic Stroke

**DOI:** 10.1155/2022/5160329

**Published:** 2022-06-29

**Authors:** Ke Song, Yikun Sun, Haoqi Liu, Yuanyuan Li, Na An, Liqin Wang, Hanlai Zhang, Fan Yang, Yanwei Xing, Yonghong Gao

**Affiliations:** ^1^Key Laboratory of Chinese Internal Medicine of Ministry of Education and Beijing, Dongzhimen Hospital Affiliated to Beijing University of Chinese Medicine, 100700 Beijing, China; ^2^Guang'an Men Hospital, China Academy of Chinese Medical Sciences, 100053 Beijing, China; ^3^Baotou Mongolian Traditional Chinese Medicine Hospital, 014040 Baotou, China; ^4^Institute of Acupuncture and Moxibustion, China Academy of Chinese Medical Sciences, 100700 Beijing, China; ^5^Institute for Brain Disorders, Beijing University of Chinese Medicine, 100700 Beijing, China

## Abstract

**Aim:**

To elucidate the mechanism of action of berberine on ischaemic stroke based on network pharmacology, bioinformatics, and experimental verification.

**Methods:**

Berberine-related long noncoding RNAs (lncRNAs) were screened from public databases. Differentially expressed lncRNAs in ischaemic stroke were retrieved from the Gene Expression Omnibus (GEO) database. GSE102541 was comprehensively analysed using GEO2R. The correlation between lncRNAs and ischaemic stroke was evaluated by the mammalian noncoding RNA-disease repository (MNDR) database. The component-target-disease network and protein-protein interaction (PPI) network of berberine in the treatment of ischaemic stroke were constructed by using network pharmacology. We then performed gene ontology (GO) and Kyoto Encyclopaedia of Genes and Genomes (KEGG) enrichment analyses. Finally, according to the molecular docking analysis and the binding probability between the lncRNA and key proteins, the effectiveness of the results was further verified by *in vitro* experiments.

**Results:**

After matching stroke-related lncRNAs with berberine-related lncRNAs, four genes were selected as potential targets of berberine in the treatment of ischaemic stroke. Subsequently, lncRNA H19 was identified as the potential crucial regulatory lncRNA of berberine. Here, 52 target proteins of berberine in the treatment of ischaemic stroke were identified through database mining. Through topological analysis, 20 key targets were identified which were enriched in inflammation, apoptosis, and immunity. Molecular docking results showed that MAPK8, JUN, and EGFR were central genes. Finally, *in vitro* experiments demonstrated that lncRNA H19, p-JNK1/JNK1, p-c-Jun/c-Jun, and EGFR expressions were significantly increased in hypoxia-treated SH-SY5Y cells and were restored by berberine treatment.

**Conclusion:**

The potential targets and biological effects of berberine in the treatment of ischaemic stroke were predicted in this study. The lncRNA H19/EGFR/JNK1/c-Jun signalling pathway may be a key mechanism of berberine-induced neuroprotection in ischaemic stroke.

## 1. Introduction

Stroke is a type of cerebrovascular disease that causes a disability and even death worldwide. Clinically, ischaemic stroke is more common than haemorrhagic stroke, accounting for 87% of all cases, and it has become the focus of most research [1]. Ischaemic stroke is caused by cerebrovascular stenosis or occlusion, and it is characterised by high complication and mortality rates [2, 3]. In recent years, with rapid economic development and population ageing, ischaemic stroke has become the fourth leading cause of death worldwide [4]. At present, the clinical treatment of ischaemic stroke mainly focuses on ultraearly thrombolysis, acute neuroprotection, and restoration of neurovascular structure and function in the recovery period. Intravenous thrombolytic therapy is the most effective method to restore blood flow within 4.5 hours after stroke [5]. However, most patients are still at risk of neurological deficits even if thrombolysis is successful. Therefore, it is urgent to find potential drugs for ischaemic stroke.

Recent studies have shown that lncRNAs, as endogenous small molecules, are extensively involved in the pathogenesis of ischaemic stroke [6–8]. A clinical study has found that the Rs217727 polymorphism of the lncRNA H19 gene is closely related to susceptibility to ischaemic stroke and can be used as a potential marker of ischaemic stroke [9]. At present, the treatment of ischaemic stroke with traditional Chinese medicine (TCM) targeting lncRNAs has also become a hotspot in the research field [10, 11]. In addition, lncRNAs regulated by berberine are involved in a variety of complex pathophysiological processes, including inflammation, oxidative stress, and apoptosis [12, 13]. All these processes may be closely related to ischaemic stroke. Therefore, it is reasonable to expect that berberine-regulated lncRNAs may play a crucial part in ischaemic stroke. However, the related pathological mechanism is not clear.

Berberine, a natural isoquinoline alkaloid extracted from *Coptis chinensis*, *Phellodendron amurense,* and other Chinese herbal medicines, possesses various biological functions [14–16]. Mounting evidence has shown that berberine can easily penetrate the blood-brain barrier (BBB) and possesses potent neuroprotective and anti-inflammatory effects against a variety of neurological disorders, such as ischaemic stroke, Alzheimer's disease, and subarachnoid haemorrhage injury [17–19]. Zhu et al. discovered that berberine may improve functional recovery and promote angiogenesis following transient middle cerebral artery occlusion via AMPK-dependent microglial M2 polarization [20]. Clinical studies have found that berberine improves the degree of neurological deficit and the prognosis of patients with acute cerebral infarction and that it has an important regulatory effect on CXCL6, IL-33, and MMP9 levels [21–23]. Recently, accumulating evidence has demonstrated that berberine has good therapeutic effects on ischaemic stroke, but the specific mechanism of berberine intervention needs to be further clarified.

In the past few years, bioinformatics and microarray techniques have been widely used to mine genetic targets for a variety of diseases to help researchers identify differentially expressed genes and potentially different signalling pathways. Based on these approaches, more lncRNAs will be discovered, which will expand our understanding of the molecular mechanisms underlying ischaemic stroke. Network pharmacology integrates the technology and content of systems biology, multidirectional pharmacology, network analysis, and other disciplines, and it systematically evaluates the interaction mechanisms between diseases and drugs [24, 25]. The main characteristics of network pharmacology include integrity and systematic interconnection, which are consistent with the overall concept of TCM, the basic characteristics of syndrome differentiation and treatment, and the concept of compatibility in TCM [26]. Network pharmacology reveals the interaction network of drugs, targets, and diseases, which aids in the preliminary understanding of the mechanism of multitarget drug treatment of complex diseases [27].

Here, to elucidate the pharmacological mechanism of berberine, we adopted a systematic method based on bioinformatics analysis, network pharmacology, and experimental verification of berberine intervention on ischaemic stroke. This approach provides an effective strategy to explore the molecular mechanism of berberine against ischaemic stroke and to identify potential protein targets with synergistic effects. A flowchart of the study is shown in Figure 1.

## 2. Materials and Methods

### 2.1. LncRNA Prediction of Berberine in Ischaemic Stroke

#### 2.1.1. Berberine-Related LncRNA Screening

As of October 20, 2021, we conducted literature searches in PubMed, EMBASE, CNKI database, and Google Scholar database to search for qualified studies detailing the biological effects of berberine-related lncRNAs in diseases. The following MeSH or free text terms were used to search the databases: (“berberine” OR “BBR”) and (“long noncoding RNA” OR “lncRNA”).

#### 2.1.2. Retrieval of Ischaemic Stroke-Related LncRNAs

Ischaemic stroke-related lncRNAs were obtained from the GEO database (https://www.ncbi.nlm.nih.gov/geo/) [28, 29]. The GSE102541 dataset comprised the lncRNA expression data of acute cerebral infarction (ACI) (*n* = 6) and healthy controls (Con) (*n* = 3), and it was processed using the GEO2R online analysis tool. The diagram was plotted by an online platform (https://www.bioinformatics.com.cn) for data analysis and visualisation. The cut-off criteria in this analysis were set as *P* value <0.05 and |log2(fold change)| >1.

#### 2.1.3. Crucial Regulatory LncRNA Involving Berberine in Ischaemic Stroke

The intersection of berberine-related lncRNAs and ischaemic stroke-related lncRNAs was visualised using an online mapping tool (https://bioinformatics.psb.ugent.be/ webtools/Venn/). MNDR is a database that curates the associations between ncRNAs and disease [30]. To further understand the relationship between lncRNAs and ischaemic stroke, we evaluated their correlation using the MNDR3.1 database (https://www.rna-society.org/mndr/home.html).

### 2.2. Prediction of Target Proteins Involving Berberine in Ischaemic Stroke

#### 2.2.1. Target Proteins of Berberine

Berberine structure information was obtained from NCBI PubChem (https://pubchem.ncbi.nlm.nih.gov/) [31]. Therapeutic target genes involving berberine in IS were acquired from the Swiss Target Prediction (http://www.swisstargetprediction.ch/) [32], SymMap (https://www.Symmap.org/) [33], Comparative Toxicogenomics Database (CTD) (https://ctdbase.org/) [34], STITCH (https://stitch.embl.de/) [35], SEA (https://sea.bkslab.org/) [36], and Targetnet (https://targetnet.scbdd.com/) [37]. STITCH selected the targets with scores ≥0.8, and Targetnet selected targets with probabilities ≥0.85 in the prediction results for further analysis. With the help of the UniProt database (https://www.UniProt.org/), the species was limited to “human” [38].

#### 2.2.2. Potential Targets in Ischaemic Stroke

All targets associated with ischaemic stroke were collected from the Therapeutic Target Database (TTD) (https://db.idrblab.net/ttd/) [39], DrugBank (https://www.drugbank.ca/) [40], GeneCards (https://www.genecards.org/) [41], and DisGeNET (https://www.disgenet.org/) [42]. After amalgamation of the targets from the four databases, Venny 2.1.0 (https://bioinfogp.cnb.csic.es/tools/venny/) was used to map the component targets of berberine to the disease targets of ischaemic stroke [43].

#### 2.2.3. PPI Data

The potential targets of berberine in the treatment of ischaemic stroke were imported into the STRING database (https://string-db.org/) [44], and the protein interaction network of the target groups was constructed. The species was set as “Homo sapiens,” and the minimum interaction threshold was set to 0.9. Cytoscape 3.8 software (https://www.cytoscape.org/) was used to draw a PPI network diagram for visual analysis [45].

#### 2.2.4. Screening of Crucial Target Proteins

Combined with the related literature and with the help of topological parameters, such as closeness centrality (Cc), eigenvector centrality (EC), network centrality (NC), local average connectivity (LAC), betweenness centrality (BC), and degree (DC), the CytoNCA network topology analysis plug-in [46] was used to further analyse the PPI network topology structure. The number of nodes was more than twice the median value of the DC and BC, and the Cc, EC, NC, and LAC nodes larger than the median value were considered to be crucial target proteins in the protein interaction networks.

#### 2.2.5. Enrichment Analysis

To further explain the role of the target proteins in the active components of TCM on gene and pathway functions, we used the DAVID database (https://david.ncifcrf.gov/) to perform GO and KEGG enrichment analyses [47]. Enrichment *P* values <0.01 were considered the screening condition to screen out the potential pathway of berberine in the treatment of ischaemic stroke.

#### 2.2.6. Molecular Docking between Target and Compound

The structure map of berberine was downloaded from the PubChem database, and the crystal structure of the key target proteins, based on DC, BC, Cc, EC, NC, and LAC, was the ligand and the core target protein was used as the receptor for molecular docking downloaded from the RCSB protein database (https://www.rcsb.org/) [48]. Berberine was used as a ligand and core target protein as a receptor for molecular docking. AutoDock tools-1.5.6 software was used for molecular docking [49]. Ligplot + v.2.2 software and Discovery Studio 4.5 were used to visualise the docking results and establish the docking interaction pattern diagram [50]. According to the docking results, the conformation with lower binding energy and better conformation was selected to evaluate the binding activity of berberine with the target protein.

### 2.3. LncRNA-Protein Interaction Prediction

We searched the nucleotide sequences of lncRNA H19 and key targets of molecular docking through the NCBI and UniProt databases. Based on the nucleotide sequence, the interaction probability between lncRNA H19 and key targets was predicted by the RNA-Protein Interaction Prediction (RPISeq) database (https://pridb.gdcb.iastate.edu/RPISeq/index.html) [51].

### 2.4. Experimental Verification

#### 2.4.1. Reagents

Sterile filtered dimethyl sulfoxide (DMSO) was obtained from Gibco (USA). Berberine was purchased from Yuanye (B21379, China) and was dissolved in DMSO [52]. Dulbecco's modified Eagle's medium (DMEM, Gibco, USA) and foetal bovine serum (FBS, Gibco, USA) were used for cell culture. Rabbit monoclonal antibodies specific for JNK1, p-c-Jun, c-Jun, EGFR, and *β*-actin were purchased from Abcam (USA), and rabbit polyclonal antibodies against p-JNK1 were purchased from Cell Signaling Technology (USA).

#### 2.4.2. Cell Culture and Treatments

Human neuroblastoma SH-SY5Y cells were obtained from the Cell Culture Centre at the Institute of Basic Medical Sciences (IBMS) of the Chinese Academy of Medical Sciences (CAMS) and cultured in DMEM containing 10% FBS in an automatic CO_2_ incubator (37°C, 5% CO_2_; Sanyo, Japan). The hypoxia model was conducted according to previous studies [53, 54]. Cells were cultured in a hypoxia (1% O_2_) condition to mimic ischaemia stroke *in vitro*. Briefly, cells were seeded at a density of 5 × 10^4^ cells/ml in culture dishes for 48 h. After reaching 80% confluence, cells were randomly divided into control group, model group, and different berberine groups. The medium was replaced by serum-free DMEM in each group. The berberine groups were treated with the final concentration of 10, 20, and 50 *μ*M, respectively, before hypoxia. The model group and different berberine groups were exposed to hypoxia in a three-gas incubator (1% O_2_; Memmert, Germany) at 37°C for 24 h. The control group was incubated in normoxic conditions for the same time. The morphology of SH-SY5Y cells in each group was observed under an inverted microscope.

#### 2.4.3. Cell Viability

Cell viability was detected by CCK8 assay according to the manufacturer's instructions. Briefly, cells were treated with berberine (10, 20, and 50 *μ*M) in the hypoxia model. After treatment, the culture medium was removed from the wells, and 10 *μ*l of CCK8 solution was added to each well in 100 *μ*l of medium followed by incubation at 37°C for 2 h. The absorbance was subsequently measured at 490 nm with a microplate reader (Thermo Scientific, USA).

#### 2.4.4. Western Blot Analysis

The concentration of protein extracted from the cells was determined by a BCA protein assay kit (Applygen, China). Equal amounts (30 *μ*g) of protein were then electrophoresed on a 10% gradient SDS‐PAGE gel and transferred to PVDF membranes (Millipore, USA). After the membranes were blocked with 5% skim milk or 5% BSA for 1 hour at room temperature, they were incubated at 4°C overnight with the following primary antibodies: JNK1 (1 : 1000), p-JNK1 (1 : 2000), c-Jun (1 : 5000), p-c-Jun (1 : 2000), EGFR (1 : 5000), and *β*‐actin (1 : 5000). The membranes were then incubated with secondary antibodies at room temperature for 1 hour. Super ECL Plus (Beyotime, China) was added to the membranes, and protein bands were visualised on a chemiluminescence imaging system (Bio-Rad, Canada). The optical density (OD) value of the protein bands was determined by ImageJ software.

#### 2.4.5. Quantitative Real-Time PCR (qRT-PCR)

Total RNA was isolated with an RNAprep Pure Cell/Bacteria Kit (TIANGEN, Biotech, China). cDNA was synthesized using FastKing gDNA Dispelling RT SuperMix (TIANGEN, Biotech, China) according to the manufacturer's instructions. qRT-qPCR was performed with an Applied Biosystems 7500 using SuperReal PreMix Plus (TIANGEN, Biotech, China). The following primers were used: lncRNA H19 forward, 5′-CGCTTTTGAACCAGCAGGG-3′; lncRNA H19 reverse, 5′-TTCCCGAGGCTTT GGTGTG-3′; GAPDH forward, 5′-GGAGTCCACTGGCGTCTTCA-3′; and GAPDH reverse, 5′-GTCATGAGTCCTTCCACGATACC-3′. GAPDH was utilized as the reference gene.

### 2.5. Statistical Analysis

Data are expressed as the means ± SD. GraphPad Prism 8.0 was utilized for visualisation of data. Differences in multiple groups were analysed by ANOVA. *P* values <0.05 were considered statistically significant.

## 3. Results

### 3.1. Retrieval of Berberine-Related LncRNAs

Using “Berberine” and “lncRNA” as the keywords for searching PubMed, EMBASE, CNKI database, and Google Scholar database, CASC2, RP5-1057I20.5, MIAT, LINC00943, BACE1-AS, LASER, MRAK052686, H19, HOTAIR, and MALAT1 were found to be associated with berberine (Table 1). Furthermore, we explored the regulatory effects of berberine on lncRNA expression and revealed the underlying molecular mechanisms. Berberine plays a role in various pathological mechanisms by regulating lncRNAs, such as inflammation, autophagy, and apoptosis.

### 3.2. LncRNA H19 Is the Crucial Regulatory LncRNA Influenced by Berberine in Ischaemic Stroke

A total of 13011 differentially expressed lncRNAs were screened from the GSE102541 dataset with 4732 upregulated genes and 8279 downregulated genes (Figures 2(a) and 2(b)). After matching ischaemic stroke-related lncRNAs with berberine-related lncRNAs (Figure 2(c)), four genes (H19, HOTAIR, CASC2, and LINC00943) were selected as potential targets for berberine in the treatment of ischaemic stroke. The heatmap of these genes is shown in Figure 2(d). To further understand the relationship between these genes and ischaemic stroke, the MNDR3.1 database was used by integrating experimentally supported and predicted ncRNA-disease associations curated from literature and other resources. As shown in Table 2, studies have shown that H19 is highly expressed in stroke patients, rat cerebral ischaemic reperfusion models, and cellular oxygen glucose deprivation/reperfusion (OGD/R) models [66, 67] with a confidence score between lncRNA H19 and ischaemic stroke >0.99, indicating that lncRNA H19 has a strong correlation with ischaemic stroke. LncRNA H19 may be the crucial regulatory lncRNA regulated by berberine in ischaemic stroke.

### 3.3. Target Proteins of Berberine in Ischaemic Stroke

For compound target identification, 422 targets of berberine were identified from the Swiss Target Prediction, SymMap, CTD, STITCH, SEA, and Targetnet databases. The 3387 targets identified in ischaemic stroke were obtained after sorting from the TTD, GeneCards, Drugbank, and DisGeNET databases. By using Venny 2.1 drawing software, 248 treatment targets were selected as potential targets of berberine in the treatment of ischaemic stroke (Figure 3(a)). A PPI network diagram of potential targets of berberine in the treatment of ischaemic stroke was generated using the STRING database. The potential targets were imported into Cytoscape software to build a compound-target-disease network diagram (Figure 3(b)). CytoNCA was used to calculate the topological parameter information, including BC, Cc, EC, LAC, NC, and DC, according to the topological attributes of the network nodes. The crucial target screening strategy is shown in Figure 3(c). The results showed that 20 target proteins, including AKT1, MAPK1, MAPK3, RELA, and TP53, were the core nodes of the entire network. The network topology parameter information of the 20 key targets of berberine in ischaemic stroke is shown in Table 3.

### 3.4. GO and KEGG Enrichment Analyses of Core Targets

In the GO enrichment analysis, 162 items were obtained from 20 core targets with a *P* value <0.01, including 117 biological process (BP) terms, 14 cell composition (CC) terms, and 31 molecular function (MF) terms. The top 10 BP, CC, and MF terms are screened and are represented by a bar chart in Figure 4(a). The protein-encoding was found to be involved in biological processes, such as positive regulation of transcription from the RNA polymerase II promoter, negative regulation of apoptotic processes, and signal transduction. The molecular functions of these proteins included protein binding, transcription factor binding, and enzyme binding. These findings suggested that berberine may have various biological functions through multiple targets to protect against ischaemic stroke. KEGG enrichment analysis identified 92 signalling pathways, and the top 20 pathways are shown in the bubble chart (Figure 4(b)). As shown in Table 4, the enrichment results demonstrated that the “MAPK signalling pathway,” “Toll-like receptor signalling pathway,” “Prolactin signalling pathway,” “TNF signalling pathway,” “ErbB signalling pathway,” and “HIF-1 signalling pathway” were closely related to the onset and progression of ischaemic stroke. These results indicated that berberine regulates multiple inflammation, immunity, metabolism, and apoptosis pathways to prevent ischaemic stroke. The details of the top 20 pathways and core targets of berberine in the treatment of ischaemic stroke are shown in Figure 5.

### 3.5. Molecular Docking

To further validate candidate berberine targets in ischaemic stroke, we tested the precision of docking between berberine and the following potential target proteins: MAPK8, JUN, EGFR, STAT3, MAPK1, SRC, MAPK14, MAPK3, AKT1, and MYC. The stable docking model has a negative binding energy, lower energy score, stronger ligand-receptor binding ability, and a more stable structure [68]. In the present study, the binding energy of berberine with 10 core targets ranged from −3.08 to −5.77 kJ·mol^−1^ (Table 5).  Figure 6 shows the following interaction points: JNK1 mainly interacted with berberine via amino acid residues Ala33, Glu58, Gly35, Lys53, Lie54, Met36, Ser55, Thr66, Tyr34, and Tyr62; JUN mainly interacted with berberine via amino acid residues Ala0, Ala4, Arg16, Asn17, He3, Glu7, Glu15, Gln12, Leu13, and Lys14; and EGFR mainly interacted with berberine via amino acid residues Asp984, Arg977, Gln974, Glu985, Gly983, He981, and Val980. These results suggested that berberine is closely bound to core target protein residues through multifaceted interactions. Overall, these results provide further evidence that these proteins act as crucial targets of berberine in the treatment of ischaemic stroke.

### 3.6. Prediction of LncRNA H19-Protein Interactions

To further investigate the potential role of lncRNA H19, we evaluated the binding probability between lncRNA H19 and key proteins through random forest (RF) or support vector machine (SVM). As shown in Figure 7, the RF and SVM between lncRNA H19 and JNK1 and EGFR were both greater than 0.5, indicating that lncRNA H19 may have a direct regulatory relationship with both JNK1 and EGFR.

### 3.7. Berberine Attenuated Ischaemic Stroke via Regulation of the LncRNA *H19/*EGFR/*JNK1/c-*Jun pathway in *SH-SY5Y* cells

To explore the neuroprotective effects of berberine by regulating lncRNA H19, we induced hypoxia injury in SH-SY5Y cells. As shown in Figure 8(a), berberine (10 and 20 *μ*M) reduced morphological damage and maintained the normal morphology of SH-SY5Y cells during cell hypoxia, and it had a significant protective effect on SH-SY5Y cell injury. The CCK8 assay indicated that cell viability was significantly enhanced after berberine treatment at concentrations of 10 *μ*M and 20 *μ*M (Figure 8(b)). According to the CCK8 experiment and cell morphology analysis, the lowest effective concentration of berberine (10 *μ*M) was selected for subsequent signalling pathway studies. The expression levels of lncRNA H19, EGFR, p-JNK1/JNK1, and p-c-Jun/c-Jun in SH-SY5Y cells were then evaluated. The results indicated that the expression levels of lncRNA H19, EGFR, p-JNK1/JNK1, and p-c-Jun/c-Jun were significantly increased in SH-SY5Y cells after hypoxia injury and were normalised by berberine treatment (Figures 8(c)–8(f)). These data suggested that berberine attenuates ischaemic stroke via regulation of the lncRNA H19/EGFR/JNK1/c-Jun pathway in hypoxia-treated SH-SY5Y cells.

## 4. Discussion

Ischaemic stroke remains a main cause of death and disability worldwide, and more effective drug treatment is urgently needed [69, 70]. Berberine is an alkaloid isolated from the Chinese herbal medicine, *Coptis chinensis*, which is widely used as a hypoglycaemic, lipid-lowering, anti-inflammatory, and anticancer drug in China [71–74]. Recent studies have demonstrated that berberine has a good effect on ischaemic stroke [20]. In the present study, we systematically revealed the protective mechanism of berberine from ischaemic stroke by means of bioinformatics analysis, network pharmacology analysis, molecular docking, and experimental verification.

This study investigated the synergistic effect of berberine on ischaemic stroke from four aspects. First, after matching stroke-related lncRNAs with berberine-related lncRNAs, four genes were selected as potential targets for berberine in the treatment of ischaemic stroke. We further evaluated their correlation using the MNDR3.1 database and found that lncRNA H19 may be the crucial regulatory lncRNA of berberine against ischaemic stroke. Second, Venny drawing software and the PPI network identified 248 treatment targets as potential targets of berberine against ischaemic stroke. The PPI network recognised MAPK8, JUN, EGFR, STAT3, MAPK1, SRC, MAPK14, MAPK3, AKT1, MYC, TP53, FOS, RELA, IL6, ESR1, TNF, CREBBP, EP300, SHC1, and RAC1 as hub genes. The PPI network revealed the interaction of berberine with ischaemic stroke-related targets and identified possible essential targets from a more detailed perspective according to the topological attributes of the network. GO and KEGG analyses illustrated that the main signalling pathways related to these targets were as follows: MAPK signalling pathway, Toll-like receptor signalling pathway, prolactin signalling pathway, TNF signalling pathway, and HIF-1 signalling pathway. These pathways are closely related to inflammation, immunity, and oxidative stress. Molecular docking analysis between the compound and targets further validated that berberine had good binding ability with these key proteins, and the JNK1/c-Jun signalling pathway may be the crucial functional pathway. Third, we evaluated the binding probability between lncRNA H19 and key proteins, and we found that lncRNA H19 may have a direct regulatory relationship with both JNK1 and EGFR. Finally, *in vitro* experiments confirmed that berberine may have a good therapeutic effect on ischaemic stroke by regulating the lncRNA H19/EGFR/JNK1/c-Jun signalling pathway.

LncRNAs have been reported to actively participate in many important biological processes through cell cycle regulation, splicing regulation, RNA degradation, gene imprinting, and chromatin remodelling [75, 76]. LncRNA H19, as a crucial member of the lncRNA family, plays an important regulatory role in the pathophysiological processes of ischaemic stroke, such as oxidative stress, the inflammatory response, apoptosis, autophagy, and neurogenesis. A recent study has demonstrated that lncRNA H19 knockdown ameliorates cell apoptosis and inflammatory cytokine concentrations by regulating the microRNA-29b/SIRT1/ PGC-1*α* axis [77]. LncRNA H19 inhibition activates the IGF1-mediated mTOR pathway and promotes axon sprouting and functional recovery [78]. Gao et al. showed that lncRNA H19 acts as a competing endogenous RNA (ceRNA) of miR-19a-3p to target PTEN, inducing oxidative stress, increasing lactate dehydrogenase levels, increasing malondialdehyde levels, and decreasing superoxide dismutase activity, thus aggravating cerebral I/R injury [79]. A clinical study has shown that the expression levels of lncRNA H19 in patients increase within the first 24 h of stroke onset, which is closely related to the rs217727 functional polymorphism [80]. These data suggest that lncRNA H19 may be a potential biomarker for the diagnosis and treatment of ischaemic stroke. In this study, the expression of lncRNA H19 in SH-SY5Y cells increased with hypoxia-induced injury.

At present, there are relatively few studies on lncRNAs in TCM. Previous studies have shown that resveratrol, curcumin, and other active components of TCM attenuate oxidative stress, inflammation, and apoptosis by regulating lncRNAs [81, 82]. Emerging evidence also suggests that berberine-regulated lncRNA H19 markedly inhibits inflammation by reducing neutrophil activation and inhibiting immune cell infiltration and inflammatory gene expression [63]. In this work, lncRNA H19 was significantly decreased after berberine treatment.

Based on molecular docking and the correlation of lncRNA H19-proteins, we investigated the role of berberine-regulated lncRNA H19 in hypoxia-induced SH-SY5Y cells, focusing on the EGFR/JNK1/c-Jun signalling pathway. EGFR activates a variety of downstream signalling pathways, such as the JNK1/c-Jun pathway and PI3K/Akt pathway, which participate in the regulation of cell proliferation, differentiation, and angiogenesis [83–85]. Studies have indicated that blockade of the EGFR pathway may attenuate reactive astrogliosis by inhibiting cell cycle progression and protect against ischaemic brain injury in rats [86]. After ischaemic stroke, the release of various inflammatory factors, increased ROS production, and endoplasmic reticulum stress stimulate the activation of JNK, which phosphorylates the downstream protein, c-Jun. The JNK1/c-Jun pathway is closely related to apoptosis, autophagy, and inflammation, and it plays an important role in various nervous system diseases [87, 88]. Under hypoxic conditions, many drugs improve SH-SY5Y cell apoptosis and autophagy by inhibiting the JNK signalling pathway [89]. In addition, related studies have demonstrated that JNK/c-Jun signalling pathway activation may regulate neuronal apoptosis, increase the permeability of the BBB, and enlarge cerebral infarction size [90]. In addition, studies have demonstrated that EGFR activates the JNK/c-Jun signalling pathway and promotes JNK/c-Jun phosphorylation, which regulates the redistribution of ZO-1 and occluding, ultimately reducing the permeability of the BBB [91]. Therefore, the EGFR/JNK1/c-Jun signalling pathway is critical to the pathological processes of ischaemic stroke. Consistent with the above findings, the expression levels of p-JNK1/JNK1, p-c-Jun/c-Jun, and EGFR were significantly increased in SH-SY5Y cells after hypoxia-induced injury and were restored by berberine treatment.

## 5. Conclusion

In conclusion, this study utilized network pharmacology, molecular docking, and bioinformatics analysis to elucidate the relationship between complex diseases, such as ischaemic stroke, and TCM intervention. We confirmed that berberine has an excellent neuroprotective effect via regulation of the lncRNA H19/EGFR/JNK1/c-Jun pathway in hypoxia-induced SH-SY5Y cell injury, making it a possible drug candidate for ischaemic stroke. This study provides a novel strategy for a comprehensive understanding of the mechanism of berberine in ischaemic stroke. However, *in vivo* experiments need to be conducted in the future to verify these results. In addition, various high-throughput sequencing screening methods, such as sequencing and proteomic analysis, should be combined with target screening to provide more reliable evidence for these screening results.

## Figures and Tables

**Figure 1:** Study flowchart. IS: ischaemic stroke; PPI: protein-protein interaction; GO: gene ontology; KEGG: Kyoto Encyclopaedia of Genes and Genomes.

**Figure 2:** Identification of differential lncRNAs and key lncRNAs. (a) Volcano plot of all the lncRNAs in GSE102541. (b) Heatmap depicting the expression levels of differentially expressed lncRNAs in GSE102541. (c) Venn diagram of differentially expressed lncRNAs in GSE102541 and berberine-related lncRNAs. (d) Clustered heatmap of overlapping lncRNAs. ACI: acute cerebral infarction; Con: control.

**Figure 3:** Target proteins of berberine in ischaemic stroke. (a) Common target network of berberine and ischaemic stroke. (b) Regulatory network of component-disease-targets. (c) Target screening strategy for key nodes in berberine. The yellow nodes represent the crucial targets of the entire network. IS: ischaemic stroke; DC: degree; BC: betweenness centrality; Cc: closeness centrality; EC: eigenvector centrality; NC: network centrality; LAC: local average connectivity.

**Figure 4:** GO and KEGG enrichment analyses for berberine in the treatment of ischaemic stroke. (a) GO enrichment analysis. (b) KEGG enrichment analysis. BP: biological process; CC: cell composition; MF: molecular function; GO: gene ontology; KEGG: Kyoto Encyclopaedia of Genes and Genomes.

**Figure 5:** Bubble map of enrichment pathways of the main targets in berberine. The red node represents the potential core target of berberine in ischaemic stroke, and the blue node represents the target-related KEGG pathway.

**Figure 6:** Structural interactions between active proteins and berberine.

**Figure 7:** LncRNA H19-protein interaction prediction. Interaction probabilities generated by RPISeq range from 0 to 1. In performance evaluation experiments, predictions with probabilities >0.5 were considered “positive,” that is, indicating that the corresponding RNA and protein are likely to interact. RF: random forest; SVM: support vector machine.

**Figure 8:** Berberine prevented ischaemic stroke by inhibiting the lncRNA H19/EGFR/ JNK1/c-Jun pathway. (a) The morphology of SH-SY5Y cells in each group was observed under an inverted microscope (scale bars: 100 *μ*m). (b) Viability of SH-SY5Y cells after berberine treatment as evaluated by a CCK8 assay (*n* = 5). (c) Validation of lncRNA H19 expression by qRT‐PCR analysis (*n* = 4-5). ((d–f)) Western blot analysis was used to detect the protein expression levels of EGFR, p-JNK1/JNK1, and p-c-Jun/c-Jun in SH-SY5Y cells (*n* = 5). Note: model versus control, ^*∗*^*P* < 0.05; berberine versus model, ^#^*P* < 0.05.

**Table 1:** Pathological mechanism of berberine-regulated lncRNAs.

LncRNA	Mechanism	Gene	Ref.
CASC2	Apoptosis	Bcl-2, Bax, Casp3, Casp9, Mcl1, Bad1, PARP2	[55, 56]
RP5-1057I20.5	Insistance	ROS	[57]
MIAT	Autophagy	p62, BNP, mTOR, AMPK, LC3	[58, 59]
LINC00943	Inflammation and cell apoptosis	KPNA4, NF-*κ*B, IL6, TNFa	[12]
BACE1-AS	Inflammation, oxidative stress, and cell apoptosis	ROS, Ca^2+^, Bcl-2, Bax, Caspase3	[60]
LASER	Cholesterol homeostasis	HNF-1, PCSK9	[61]
MRAK052686	Inflammation and oxidative stress	Nrf2	[62]
H19	Oxidative stress and inflammation	NF-*κ*B, NOX2, ROS	[63]
HOTAIR	Migration, invasion, and apoptosis	E-cadherin, vimentin, snail	[64]
MALAT1	Inflammation	IL6, IL1*β*, TNF*α*, IL10	[65]

**Table 2:** Correlation predictions between lncRNAs and ischaemic stroke.

LncRNA	Disease name	LncRNA expression	Evidence support	Confidence score	PubMed ID
H19	Ischaemic stroke	Upregulated	ELISA//flow cytometry//IF//qRT-PCR//western blot	0.999999	28630232
H19	Cerebral ischaemia-reperfusion injury	Upregulated	Cell transfection//cell viability assay//flow cytometry//IF//qRT-PCR//western blot	1	28203482
CASC2	Brain ischaemic	N/A	Computational predicted	0.073106	N/A
LINC00943	N/A	N/A	N/A	N/A	N/A
HOTAIR	Brain ischaemic	N/A	Computational predicted	0.073106	N/A

**Table 3:** Network topology parameter information of 20 key targets of berberine in the treatment of ischaemic stroke.

Swiss-Prot	Genes	Description	Validated or predicted	BC	Cc	EC	LAC	NC	DC
P45983	MAPK8	Mitogen-activated protein kinase 8	Predicted	1.77	1	0.23	16.84	19	19
P05412	JUN	Transcription factor AP-1	Predicted	1.77	1	0.23	16.84	19	19
P00533	EGFR	Epidermal growth factor receptor	Validated	1.77	1	0.23	16.84	19	19
P40763	STAT3	Signal transducer and activator of transcription 3	Predicted	1.77	1	0.23	16.84	19	19
P28482	MAPK1	Mitogen-activated protein kinase 1	Validated	1.77	1	0.23	16.84	19	19
P12931	SRC	Proto-oncogene tyrosine-protein kinase Src	Predicted	1.77	1	0.23	16.84	19	19
Q16539	MAPK14	Mitogen-activated protein kinase 14	Validated	1.77	1	0.23	16.84	19	19
P27361	MAPK3	Mitogen-activated protein kinase 3	Predicted	1.77	1	0.23	16.84	19	19
P31749	AKT1	RAC-alpha serine/threonine-protein kinase 1	Validated	1.77	1	0.23	16.84	19	19
P01106	MYC	Myc proto-oncogene protein	Predicted	1.77	1	0.23	16.84	19	19
P04637	TP53	Cellular tumour antigen p53	Validated	0.57	0.95	0.23	16.56	17.88	18
P01100	FOS	Proto-oncogene c-Fos	Predicted	0.57	0.95	0.23	16.56	17.88	18
Q04206	RELA	Transcription factor p65	Validated	1	0.95	0.22	16.33	17.76	18
P05231	IL6	Interleukin-6	Predicted	0.57	0.95	0.23	16.56	17.88	18
P03372	ESR1	Oestrogen receptor	Predicted	0.57	0.95	0.23	16.56	17.88	18
P01375	TNF	Tumour necrosis factor	Predicted	1	0.95	0.22	16.33	17.76	18
Q92793	CREBBP	CREB-binding protein	Predicted	0	0.90	0.22	16	17	17
Q09472	EP300	Histone acetyltransferase p300	Validated	0	0.90	0.22	16	17	17
P29353	SHC1	SHC-transforming protein 1	Validated	0	0.79	0.18	13	14	14
P63000	RAC1	Ras-related C3 botulinum toxin substrate 1	Predicted	0	0.73	0.15	11	12	12

**Table 4:** List of enrichment pathways of the main targets of berberine.

Gene-pathway network	No. of genes	Fold enrichment	*P* value	Bonferroni method	Gene names
Hepatitis B	15	35.58103448	1.91*E* − 20	2.72*E* − 18	CREBBP, JUN, SRC, STAT3, FOS, TNF, RELA, IL6,MAPK8, MYC, AKT1, EP300, MAPK1, TP53, MAPK3
Prolactin signalling pathway	11	53.28802817	6.06*E* − 16	7.88*E* − 14	MAPK8, SHC1, SRC, STAT3, MAPK1, AKT1, FOS, MAPK14, ESR1, RELA, MAPK3
Pathways in cancer	15	13.1278626	2.82*E* − 14	4.00*E −*12	CREBBP, JUN, STAT3, FOS, EGFR, RELA, IL6, MAPK8, MYC, AKT1, EP300, MAPK1, RAC1, TP53, MAPK3
Toll-like receptor signalling pathway	11	35.69292453	4.03*E* − 14	5.72*E* − 12	IL6, JUN, MAPK8, MAPK1, AKT1, FOS, RAC1,MAPK14, TNF, RELA, MAPK3
MAPK signalling pathway	13	17.67332016	1.90*E* − 13	2.70*E* − 11	JUN, FOS, MAPK14, TNF, EGFR, RELA, MAPK8, MYC, AKT1, MAPK1, RAC1, TP53, MAPK3
Proteoglycans in cancer	12	20.637	5.89*E* − 13	8.36*E* − 11	SRC, MYC, STAT3, MAPK1, AKT1, RAC1, MAPK14, ESR1, TNF, TP53, EGFR, MAPK3
Colorectal cancer	9	49.92822581	1.91*E* − 12	2.71*E* − 10	JUN, MAPK8, MYC, MAPK1, AKT1, FOS, RAC1, TP53, MAPK3
Chagas disease (American trypanosomiasis)	10	33.07211538	2.37*E* − 12	3.36*E* − 10	IL6, JUN, MAPK8, MAPK1, AKT1, FOS, MAPK14, TNF, RELA, MAPK3
Pancreatic cancer	9	47.62384615	2.84*E* − 12	4.03*E* − 10	MAPK8, STAT3, MAPK1, AKT1, RAC1, TP53, RELA, EGFR, MAPK3
TNF signalling pathway	10	32.14485981	3.08*E* − 12	4.37*E* − 10	IL6, JUN, MAPK8, MAPK1, AKT1, FOS, MAPK14, TNF, RELA, MAPK3
Influenza A	11	21.74396552	6.29*E* − 12	8.93*E* − 10	IL6, CREBBP, JUN, MAPK8, EP300, MAPK1, AKT1, MAPK14, TNF, RELA, MAPK3
Tuberculosis	11	21.37542373	7.47*E* − 12	1.06*E* − 09	IL6, CREBBP, MAPK8, SRC, EP300, MAPK1, AKT1, MAPK14, TNF, RELA, MAPK3
Neurotrophin signalling pathway	10	28.6625	8.82*E* − 12	1.25*E* − 09	JUN, MAPK8, SHC1, MAPK1, AKT1, RAC1, MAPK14, TP53, RELA, MAPK3
Pertussis	9	41.274	9.36*E* − 12	1.33*E* − 09	IL6, JUN, MAPK8, MAPK1, FOS, MAPK14, TNF, RELA, MAPK3
Osteoclast differentiation	10	26.25572519	1.97*E* − 11	2.79*E* − 09	JUN, MAPK8, MAPK1, AKT1, FOS, RAC1, MAPK14, TNF, RELA, MAPK3
*Salmonella* infection	9	37.29578313	2.16*E* − 11	3.07*E* − 09	IL6, JUN, MAPK8, MAPK1, FOS, RAC1, MAPK14, RELA, MAPK3
Hepatitis C	10	25.86090226	2.26*E* − 11	3.20*E* − 09	MAPK8, STAT3, MAPK1, AKT1, MAPK14, TNF, TP53, RELA, EGFR, MAPK3
FoxO signalling pathway	10	25.66791045	2.42*E* − 11	3.43*E* − 09	IL6, CREBBP, MAPK8, STAT3, EP300, MAPK1, AKT1, MAPK14, EGFR, MAPK3
ErbB signalling pathway	9	35.58103448	3.18*E* − 11	4.52*E* − 09	JUN, MAPK8, SHC1, SRC, MYC, MAPK1, AKT1, EGFR, MAPK3
HIF-1 signalling pathway	9	32.2453125	7.13*E* − 11	1.01*E* − 08	IL6, CREBBP, STAT3, EP300, MAPK1, AKT1, RELA, EGFR, MAPK3

**Table 5:** The results of molecular docking analysis.

Target name	PDB ID	Drug	Main binding sites with the amino acid	Binding energy (kJ/mol)
MAPK8	2OJG	Berberine	ALA-33, TYR-34, GLY-35, MET-36, LYS-53, ILE-54, SER-55, GLU-58, TYR-62, THR-66	−5.77
EGFR	5GNK		GLN-976, ARG-977, VAL-980,ILE-981, GLY-983, ASP-984, GLU-985	−5.53
SRC	4MXO		CYS-483, PRO-484, PRO-485, GLU-486, CYS-487, PRO-488, GLU-489, TYR-527, GLN-528,	−4.87
JUN	5FV8		ALA-0, ILE-3, ALA-4, GLU-7, GLN-12, LEU-13, LYS-14, GLU-15, ARG-16, ASN-17	−4.43
MAPK14	3KF7		HIS-228, HE-229, SER-254, ASN-257, TYR-258, LEU-195	−4.14
AKT1	3MVH		SER-378, SER-381, LYS-385, GLY-382, LEU-392, GLU-401, GLN-404, ARG-406	−4.03
MAPK3	4QTB		LFU-93, ILE-103, ARG-370, PHE-371	−3.86
MAPK1	5BUJ		ARG-89, PHE-346, GLU-347, ALA-350, GLN-353, PRO-354, GLY-355, TYR-356	−3.74
STAT3	4E68		DT-1001, DG-1002, DC-1003, DA-1004	−3.6
MYC	6G6K		HIS-207, LEU-951, GLN-954, GLA-955, GLN-958, LYS-959, SER-962	−3.08

## Data Availability

The data used to support the findings of this study are available from the corresponding author upon reasonable request.

## Abbreviations

GEO: Gene Expression Omnibus
MNDR: Mammalian noncoding RNA-disease repository
PPI: Protein-protein interaction
GO: Gene ontology
KEGG: Kyoto Encyclopaedia of Genes and Genomes
TCM: Traditional chinese medicine
BBB: Blood-brain barrier
IS: Ischaemic stroke
ACI: Acute cerebral infarction
Con: Control
CTD: Comparative toxicogenomics database
TTD: Therapeutic target database
Cc: Closeness centrality
EC: Eigenvector centrality
NC: Network centrality
LAC: Local average connectivity
BC: Betweenness centrality
DC: Degree
DMSO: Dimethyl sulfoxide
DMEM: Dulbecco's modified Eagle's medium
FBS: Foetal bovine serum
IBMS: Institute of Basic Medical Sciences
CAMS: Chinese Academy of Medical Sciences
qRT-PCR: Quantitative real-time PCR
OGD/R: Oxygen glucose deprivation/reperfusion
BP: Biological process
CC: Cell composition
MF: Molecular function
RF: Random forest
SVM: Support vector machine
CeRNA: Competing endogenous RNA.
